The article "Evidence-based support for S1 transpedicular screw entry point modification" was published in 2014. Journal: J Orthop Surg Res.

# Evidence-based support for S1 transpedicular screw entry point modification

**DOI:** 10.1186/1749-799X-9-22

**Published:** 2014-04-03

**Authors:** Lukasz Kubaszewski, Andrzej Nowakowski, Jacek Kaczmarczyk

**Affiliations:** 1 Department of Orthopaedic and Traumatology, W. Dega University Hospital, University of Medical Science Poznan, 28 Czerwca 1956 r Street, Poznań 61-545, Poland; 2 Spine Surgery Oncological Orthopaedic and Traumatology Department, W. Dega University Hospital, University of Medical Science Poznan, 28 Czerwca 1956 r Street, Poznań 61-545, Poland

**Keywords:** Surgical technique, Transpedicular stabilization, Spine, Sacrum, Spinal fusion, Anatomy

## Abstract

**Background:**

In the literature, ‘below and lateral to the superior S1 facet’ is defined as the basic technique for screw introduction. Until a recently published modification, no analysis for alternative starting point has been proposed nor evaluated, although some surgeons claim to use some modifications. In this study, we analyse the data from anatomical and radiological studies for optimal starting point in transpedicular S1 screw placement.

**Methods:**

A Medline search for key word combination: sacrum, anatomy, pedicle, screws and bone density resulted in 26 publications relevant to the topic. After a review of literature, two articles were chosen, as those including the appropriate set of data. The data retrieved from the articles is used for the analysis. The spatial relation of S1 facet, pedicles and vertebral body with cortical thickness and bone density in normal, osteopenic and osteoporotic sacrum is analysed.

**Results:**

Presented data advocates for more medial placement of the screws due to higher bone density and lower bone loss in osteoporosis. Medial shift of the starting point does not increase the risk of spinal canal perforation. Osteoarthritic changes within the facet can augment the posterior supporting point for screw. The facet angular orientation is similar to convergent screw trajectory.

**Conclusions:**

Modified technique for S1 screw placement takes advantage of latest anatomical and clinical data. In our opinion, technique modification improves the reproducibility and may increase stability and the screws within the posterior cortex of the S1 vertebra. Further biomechanical and clinical study should be performed to prove its superiority to classical technique.

## Background

The lumbosacral junction is the anatomical region where degeneration changes of the spine are most often observed. One of the theories which justifies the above is the biomechanical analysis, making junction of mobile lumbar spine and immobile sacrum responsible for acceleration of degenerative process. Another factor aggravating the local biomechanics is spatial configuration, causing shear forces, whose effects are best seen in spondylolisthesis [1].

Stabilization procedures extending fusion over the lumbosacral junction is usually performed in treatment of degenerative disc disease, degenerative scoliosis, spondylolisthesis, neoplastic lesions and trauma. Operative stabilization of the lumbar-sacral junction is associated with risk of complications such as non-union and pseudarthrosis. These complications are most often secondary to cortical fracture of the sacrum around the screws, or pullout of screws [2]. It is less likely that the cause of complications is fracture of rods or screws. Reoperation performed in such cases entails a technically demanding procedure. The risk of complications was observed in a very high percentage of cases: up to 70% [3]. Cortical fracture of the sacrum usually observed shortly after the initial surgery (on average after 42 days) and in presented series involved only women [4]. In order to avoid complications of this type, primary stabilization to the S2 vertebra or iliac bones can be performed [5,6], with optional interbody fusion from variable approaches [7,8], as well as using less common techniques with facet screws [9].

Despite the above-mentioned modification, the major supporting point is the screws in the S1 vertebrae. There are two major types of techniques for introducing screws in S1 vertebra: converging midsacral or medial (most often used) and laterally directed that may be used as a salvage option [10].

The first one was initially described by Roy-Camill et al. in 1986 [11]. The authors have proposed to enter the screws on the lateral aspect of the S1 facet. Smith et al. [12] and Carlson et al. [13] modified the technique, where the starting point of the screw was 2 mm lateral to and below the lower end of the S1 facet joint. Over time, this part of the technique has not evolved significantly [14-16], also there were no new studies confirming or reviewing this technique.

The main drawback of the technique is poor definition of the starting point. Definition such as ‘lateral aspect of the facet joint’ as well as ‘2 mm lateral to and below the lower end of the S1 facet joint’ is not precise. Facet joint, per continuum, turns into the posterior cortex of the sacrum with interindividual existence of defined border of the facet represented by the fold of the cortex.

Recently published technical note describes modified medial entry point located at the rim of the S1 facet [17]. In personal communication, some spine surgeons confirm using the above-mentioned modification, though, to the best of our knowledge, there is no literature trace of its anatomical justification and biomechanical analysis. In our paper, we intend to analyse the safety and legitimacy of the modification based on anatomical data available in the literature.

### Modification of the starting point for S1 transpedicular screw: summary

In the reviewed modification, a starting point for transpedicular screw introduction is, in comparison to classical method, more cranial and medial. The screw enters S1 through the superior facet at the rim of the articular surface after its osteotomy (Figure 1A,B,C). The hollow for screw insertion at the posterior cortex is limited from the bottom and lateral aspects by cortical layer, forming inferior pole of S1 superior facet, with natural, saddle-shaped support for transpedicular screw.

**Figure 1:** **Modified transpedicular screw starting point for S1 vertebra. (A)** Cutting line of osteotomy drawn on inferior L5 articular process. **(B)** Osteotomy site of S1 articular process margin. Posterio-lateral margin is divided into upper and bottom halves. The osteotomy is performed at the upper part of the bottom half of S1 superior articular process. **(C)** The starting point within the osteotomy site of the superior S1 facet (*x*). The screw is gaining the saddle-like support in the inferior pole **(b). (a)** Resected inferior L5 facet.

## Methods

A Medline search (January 2013) of the English language literature from 1990 through 2010 was performed using the two sets of key words (set one: sacrum, anatomy, pedicle and screws; set two: sacrum and ‘bone density’). Submitting the query resulted in 54 and 56 items for both sets, respectively. The preliminary 44 articles for set 1 and 40 for set 2 were rejected as not relevant to the topic based on the abstract revision. The remaining 10 for set 1 and 16 for set 2 articles were retrieved in full text version. None of the full text reviewed described the operative technique modification for the S1 screw placement resembling the one above [17]. After revision by coauthors, for the purpose of the study, two publications were selected, upon their consent, as comprising the appropriate set of data for analysis. The first one published by Arman et al. in 2009 deals with sacral anatomy, focusing on spine surgery application [18]. The second one published by Richards et al. (‘Bone density and cortical thickness in normal, osteopenic, and osteoporotic sacra’) gives the crucial data for quality of bone across the sacrum in both normal, osteopenic and osteoporotic bone [19].

The spatial relation of S1 facet, pedicles and vertebral body with cortical thickness and bone density in normal, osteopenic and osteoporotic sacrum was analysed. We have analysed the imposition and inclination of the facets with respect to pedicles with risk estimation for violation of the medial cortex and spinal canal penetration. Further analysis of facet orientation is correlated with optimal screw trajectory. Finally, bone mineral density and cortical thickness are referred to the modification of transpedicular screw entry point on the posterior cortex of the S1 vertebrae.

## Results

### S1 pedicles

For the posterior pedicle height, measured between the first posterior sacral foramen and superior border of the sacrum, the mean value is 20.98 ± 2.34 (all distance measurements in mm). There is no data regarding the width of the S1 pedicle. The pedicle in the sacral vertebra is not a clearly defined space, contrary to lumbar, thoracic or cervical ones, because it extends into sacral ala laterally. We may presume its width, knowing the diameter of adjacent posterior sacral foramina which for the first one is 8.14 ± 1.97 and decreases with each segment. The mean height of the S1 facet joint is 14.62 ± 1.83. Its mean width is 16.37 ± 2.14. As we see, the height of the S1 superior facet joint is smaller than the height of the pedicle. We cannot compare the width of the facet and pedicles due to undefined width of the S1 pedicle. The pedicle of S1 can be mostly defined by its medial margin which is the lateral border of the spinal canal, and this relation will be discussed later. For the median trajectory of the screw placement, the important information is the S1 vertebral body height and transverse diameter which are 30.22 ± 2.35 and 49.40 ± 5.89, respectively.

### S1–spinal canal

In operative anatomy of S1, we need to be aware of two values:

– transverse diameter of the spinal canal at the superior aperture of the sacrum (31.31 ± 3.16) and

– distance between the S1 facet joints (25.68 ± 3.80).

Particular landmark relation is presented in Figure 2, for better understanding of clinical anatomy.

**Figure 2:** **S1 anatomic landmark analysis.** The projection of the anatomical landmarks over S1 vertebral body silhouette (the notation of landmarks are the same as in the source article [17]). *r*, vertebral body transverse diameters; *v*, transverse diameter of the spinal canal at the superior aperture of the sacrum; *p*, distance between the S1 facet joints; *o*, width of the S1 facet joint; *n*, height of the S1 facet joint; *h*, distance between the first posterior sacral foramen and superior border of the sacrum (posterior pedicle height); *s*, height of the S1 vertebral body.

As for projections of the facet joints over the pedicles, we assume that

– from the anatomical observation, the centres of the facet joints are positioned slightly cranial in relation to centre of the pedicles

– from the anatomical analysis, the centres of the facet joints are more medial than centre of pedicles (values *p* vs. *v* on Figure 2).

There is hardly any risk that the centres of the facets (42.05 ± 5.94) will ever overlap the spinal canal in the frontal plane, with lateral rim of the joint surface, for the entry point, placed even more lateral.

When projecting the pedicles and joints over the vertebral body,

– the pedicles on both sides overlap the vertebral body at an average of (*r* − *v*) / 2 = 9.045 mm,

– the facet joints overlap the vertebral body at average (*r* − *p*) / 2 = 11.86 mm,

– approximately 13.63 mm ({[*p* + 2*o*] − *v*} / 2) of each lateral part of the facet joint overlaps the pedicle,

– lateral margin of the S1 facet joint falls approximately 4.58 mm ({[*p* + 2*o*] − *r*}2) laterally over the lateral margin of the vertebral body.

Starting at the lateral margin of the facet still forces the surgeon to hold the convergent trajectory for maximum screw length. However, the convergence angle will be smaller compared to the more lateral starting point. The angle will inversely depend on distance between the starting point and entrance to the vertebral body. Performing the osteotomy of the facet lateral rim decreases the distance, enabling more convergent screw introduction.

### Angles of both facet joints and transpedicular screw trajectory

The angles of both facet joints and screw trajectory were measured in relation to sagittal plane. S1 facet angle on the right-hand side is slightly higher compared to that of the left (35.71° ± 9.59° and 34.70° ± 9.66°, respectively). Pedicle screws in the anteromedial trajectory, measured by the authors, are 35.20° ± 9.62° and 33.80° ± 4.34° for the right- and left-side, respectively.

When we look at the trajectory separately for both sides, a difference is more visible on the left side, compared to the right side (31.95° ± 3.95° and 35.65° ± 4.73°, respectively). Theoretically, the worst anatomical discrepancy between the facet and screw trajectory can be expected on the left side. The maximal difference between the facet and ideal screw angles may reach 16.36° on the left side and 14.44° on the right side.

### Cortical thickness and bone mineral density of the sacrum

Cortical bone thickness in the anterior medial part of the S1 body is 2.01 mm; moving more lateral, it falls down to 1.58 mm in the para-medial region and in proximity to the sacro-iliac joint is 1.32 mm in average. The posterior cortex closest to facet joint is 1.23 mm thick. Close to the sacro-iliac joint, it is only 1.13 mm. With bone mass loss, the thickness of the cortex closest to facet joint decreases in osteopenia and osteoporosis, respectively, at 1.15 and 0.86 mm.

In contrast, the anterio-medial cortex, at the place where the tip of the transpedicular screws anchors, is observed to be thicker in patients with osteoporosis (2.32 mm). It is probably caused by the degeneration process of the region of anterior longitudinal ligament and spurs formation. There was no evaluation of the cortex within the facet joint itself, but based on the above-mentioned clinical observation, we can assume that also in degenerative process, cortical thickness within the facet joint will tend to increase despite the global bone mineral density (BMD) loss.

Mineral density of the trabecular bone, on the transverse section of the sacral bone, is highest on the line spanning between the facet joint and the anterio-medial cortex, just laterally to the spinal canal. Its density in different places starting from the posterior cortex has BMD subsequent values of 128.14, 75.12, 185.79 and 167.86 g/cm^3^. Moving more laterally, the BMD drops significantly; measured in three areas, starting from the posterior cortex, it has a value of 61.46, 31.33 in the middle and 81.76 in the area adjacent to the anterior cortex. In the analysis of Richards et al. [19], this is the region mostly endangered by BMD loss. In patients with osteoporosis, BMD values drop to 11.70, −21.46 and −1.33 g/cm^3^, respectively.

In the lateral region of the sacral ala, the BMD is 132.62 g/cm^3^ and is not as much affected by osteopenia or osteoporosis as in the middle and medial region. In the medial region, the mostly affected area is closest to the posterior cortex. Regular BMD of 128.14 g/cm^3^ drops down to 125.43 g/cm^3^ in osteopenia and is as low as 45.42 g/cm^3^ in case of osteoporosis.

## Discussion

In concluding the above analysis, we may state that

1. the posterio-lateral margin of the facet joint falls within the potential and safe area for transpedicular screw placement,

2. the angles of both facet joints and transpedicular screw trajectory, in S1 vertebra, are very similar,

3. both BMD and cortex thickness is highest in the area close to the midline anteriorly and to the facet joint posteriorly. Also, as for the quality of bone in this area, it is relatively good even in osteopenia and osteoporosis cases,

4. degenerative changes, both in the anterior cortex of the S1 body and in the area of the facet joint, should be taken into account in screw placement technique.

The comparison of the classical and evaluated techniques is summarized in the Table 1.

**Table 1:** Comparison of the classical and evaluated techniques

	**Classical technique**	**Evaluated technique**
Preparation	No particular preparation technique	Preparing osteotomy
Entry point landmarks	Not precisely defined	Clearly defined
Individual interpretation at the entry point definition	Possible	Less likely
Technical difficulty	More lateral exposure of the sacrum and soft tissue traction	Less extensive lateral exposure demanded and soft tissue traction
Screw trajectory definition in the operating field	Information cannot be drawn from local anatomy	After osteotomy, S1 facet orientation is close to optimal screw trajectory
Ultimate screw trajectory	Optimal	Possible to be less convergent
Cortical bone thickness in normal, osteopenic and osteoporotic bone	Decreasing lateralward	Higher compared to lateral position
BMD values in normal, osteopenic and osteoporotic bone	Decreasing lateralward	Higher compared to lateral position
Implantation in degenerated spine	No particular advantage	Potential increase of the cortical thickness due to the proximity of the degenerated facet and spurs formation

The better stability of the medially introduced screws can be achieved by perforation apex of the sacral promontory [20] or even through superior endplate [21]. The major drawback of the S1 vertebra anatomy is that in contrast to lumbar pedicle where the diameter is close to the diameter of the screws used as standard, allowing to get an additional point of support outside the cortex, the pedicles here are much wider than the diameter of the pedicle screw [22]. That is the reason why both cortices are crucial in achieving proper stabilization.

Some similarities to the evaluated technique modification, in the lumbar region, have been mentioned by Fuentes et al. in the mid-1980s; they wrote about ‘…small 5 millimeters resection of the inferior articular process allows a more cranial drill-hole which is more steady in the pedicle of the vertebra as confirmed by X rays controls and anatomic specimens’ [23], though this solution never has been applied for S1.

According to the data summarized above, cranial and medial shift of the starting point for the S1 screw introduction is safe because it still falls within the pedicle projection with no significantly greater risk for collision with neural structures. More medial position of the screw makes its trajectory through the highest density of the trabecular bone and region where bone loss is significantly lower in osteoporotic patients, compared to more lateral regions. Additionally, changes related to osteoarthritis of the facet can be used to augment the posterior cortex supporting point, and the saddle-like shape of the lower pole of the opening in the posterior cortex should give better support than with flat cortex perforation.

From the clinical point of view, comprehension of the angular configuration of the facet may help in taking the decision for ultimate screw trajectory for medial placement. From the practical point of view, compared to the classical technique, the modified technique gives a well-defined starting point for screw insertion, decreasing variability between surgeons and improving teaching procedure. To confirm the above data correlation, biomechanical and clinical studies have to be performed to prove its superiority to classical technique.

## Conclusions

Modification of the starting point for S1 transpedicular screw placement is justified by the analysis of available literature data. The upward and medial shift of the entry point from ‘below and lateral to the inferior tip of the superior S1 facet’ to the ‘lateral rim of the upper facet’ does not impose greater neurological risk, and the screw passes through the bone of higher durability. Additionally, BMD loss in osteoporotic patient may be compensated by osteoarthritic changes of the facets.

## Competing interests

The authors declare that they have no competing interests.

## Authors’ contributions

LK initiated the concept of the study, made literature review and analysis, and prepared the paper. AN analysed the literature and wrote and approved the final manuscript. JK accepted the concept, analysed the data and did the preliminary manuscript approval. All authors read and approved the final manuscript.
